This article has been retracted.

# Colon cancer-induced interleukin-35 inhibits beta-catenin-mediated pro-oncogenic activity

**DOI:** 10.18632/oncotarget.22857

**Published:** 2017-12-01

**Authors:** QiangYue Jiang, Lingyan Ma, RuiChao Li, JianHai Sun

**Affiliations:** ^1^ Department of Gerontology, Tongji Hospital, Tongji Medical College, Huazhong University of Science and Technology, Wuhan, Hubei Province, China; ^2^ Department of Oncology, the Third People’s Hospital, Wuhan, Hubei Province, China

**Keywords:** colon cancer, IL-35, β-catenin, inhibition, metastasis

## Abstract

The occurrence and development of colon cancer is closely related to inflammation. Therefore, this study was conducted a current retrospective research to study the effect of IL-35 (interleukin 35), a newly identified anti-infective factor, on colon cancer development. The expression of IL-35 in colon cancer samples and their adjacent normal mucosa by real-time PCR, ELISA (enzyme-linked immunosorbent assay). The effect of IL-35 on patient survival, colon cancer progression, and its effect on Wnt/β-catenine signaling pathway was also assessed. IL-35 is minimally expressed in colon cancer tissues but is highly expressed in adjacent normal tissues. The down-regulation of IL-35 was significantly associated with the American Cancer Joint Committee stage and overall survival of colon cancer patients. The overexpression of IL-35 in colon cancer cells inhibits cell migration, invasion, proliferation, colony formation and cancer stem cells by inhibiting beta-catenin. IL-35 inhibits colon neoplasms in mouse. Our results suggest that IL-35 has an inhibitory effect on the development of colon cancer as a novel prognostic indicator and potential therapeutic target.

## INTRODUCTION

Colon cancer is a common malignant tumor of the digestive tract system, of which the incidence is particularly high people of age from 45 to 51 years. During the past two decades in China, especially in large cities, the incidence rate has been increasing significantly, and colon cancer is higher than the trend of rectal cancer. In the United States, there are about 15 million people who get colon cancer each year, representing 15% of all patients diagnosed with cancer, without gender difference [1]. Since 1993, Cohen reported that the five-year survival rate of colon cancer was 54%. Although the treatment continues to improve, the 5-year survival rate has not improved significantly [2]. Due to the rapid progress of molecular biology theory and technology, monumental strides forward have been achieved in the field of biomedicine, and the research results have been applied to the field of clinical treatment [3].

Immune gene therapy focuses on strengthening the immunogenicity of tumor cells or immune response to the maglignance in human body, thereby killing the tumors endogeneously [4]. Multiple lines of evidence have shown that cytokines, such as interleukin 2 (IL-2), has a significant inhibitory effect on the tumor [5]. With the use of retrovirus as a carrier gene transfer technology, different cytokines or immune-related antigen into tumor cellscan be transducted in to cells, which injected to animal models, inducing and enhancing the anti-tumor immune function of animals. Currently, the underlying mechanism of it have been revealed. Firstly, tumor cells in autocrine form stable secretion of cytokines to activate production of cytotoxic T cells, NK cells and associated anti-tumor factors. Hosenberg experiments showed that every 24 hours, infiltrating lymphocyte (TIL) transfected with tumor necrosis factor (TNF) gene secreted TNF up to 231∼720pg/10^6^ cells, around 14 to 24 times of non-transfected gene cells [6]. Secondly, the expression of cytokine gene and co-stimulatory molecule gene in tumor cells increased the ability of antigen presentation, enhanced the expression of tumor-specific antigen, thereby stimulating the immune system to recognize tumor antigen, which resulted in anti-tumor effect. Specific and lasting anti-tumor immunity can prevent the metastasis and recurrence of malignancies. In recent years, IL-35 has been found to be a new member of the γc family, which is mainly produced by activated CD4 + T cells, can induce the differentiation of Th cells, and promote the proliferation and differentiation of T cells, NK cells as well as interferon gamma (IFN-γ), producingcytotoxic T lymphocyte (CTL) effect [7, 8]. *in vitro* studies have shown that colon cancer cells transfected with IL-35 gene can significantly inhibit the growth of colon cancer cells. Therefore, in the treatment of malignant tumors, IL-35 is considered to be one of the most promising candidates.

However, a crucial risk factor is that the transfected tumocells maintain a certain degree of tumorigenicity. Therefore, tumor can also be induced during treatment, compounding on the difficulties of elimination of tumor cells. In recent years, the more autologous tumor vaccine is to take peripheral blood mononuclear cells from the patiens, and incubate then with a fusion protein composed of recombinant prostate acid phosphate and granulocyte-macrophage colony-stimulating factor [9]. Recently, a phase III clinical trial revealed that standard interleukin 2 (IL-2) as adjuvant for tumor vaccine in III/IV melanoma achieved substantially improved outcome [10]. By carrying new genes to tumor cells after treatment of lesions or subcutaneous injection, the humoral, cellular and innate immune systems of the patients can be stimulated to kill tumor cells. The combination of both can effectively eliminate the potential risk of transfection of cytokines in the treatment of malignant tumors [11–13].

The purpose of this study is to analyze the relationship between the level of IL-35 in patients with colon cancer and the correlation between clinical factors, identify the correlation between IL-35 expression and survival rate, explore the changes of biological characteristics of colon cancer cells transfected with IL-35 gene, and provide a theoretical basis for evaluating the feasibility of preparing autologous tumor vaccine for the future colon cancer gene immunotherapy.

## RESULTS

### Decreased IL-35 expression in colon cancer biopsies

Of the 141 patients with colon cancer, 59 had no lymph node metastasis after surgery, 55 had different degrees of lymph node metastasis, and 4 had poorly differentiated adenocarcinoma. Although preoperative imaging and intraoperative exploration were diagnosed as liver multiple metastases, the area of lymph nodes were not found to metastasize [14]. A total of 1720 lymph nodes were removed from 141 patients, of which 403 were metastatic lymph nodes with a total metastasis rate of 23.4%. The levels of IL-35 and IFN-γ in the serum of the metastatic group were 1753 ± 153pg/ml and 510 ± 62pg/ml, respectively. The levels of IL-35 and IFN-γ in the serum of the non-metastatic group were 1521 ± 132pg/ml and 730 ± 85 pg/ml, respectively [15-16]. Serum IL-35 in patients with lymph node metastases were significantly lower (p=0.0348) (Figure 1).

**Figure 1:** The concentration of IL-35 in the serum of colon cancer patient of different regional lymph node metastasis degree

Similarly, the expression of IL-35 in early and late stage colon cancer was lower than that in adjacent tissues (Figure 2, p=0.00872) and the positive expression rate of IL-35 in cancer tissues with advanced stages were higher in early tumor tissues than advanced stage cancer tissue. (Table 1, p=0.0457).To investigate if IL-35 expression is correlated with survival rate, Kaplain-Meier survival analysis patients whose colon tumor tissues were with high IL-35 expression and low IL-35 expression, respectively. The survival rate of high IL-35 exprssion patients is significantly higher than that of low IL-35 expression (Figure 3, p=0.0346 by Mantel–Cox test).

**Figure 2:** Immunohistochemical map of IL-35 in colon cancer tissues and adjacent tissues (SP, ×200) **(A)** the expression of IL-35 in adjacent normal tissues; **(B)** the expression of IL-35 in early stage of colonrectal carcinoma; **(C)** the expression of IL-35 in middle stage of colonic carcinoma; **(D)** the expression of IL-35 at the late stage of colon carcinoma.

**Table 1:** The expression of IL-35 in different stages of colon cancer and adjacent tissues

Group	Number of cases	IL-35			IL-35 Positive expression rate/%
		—	+	++	
Early group	73				
Tumor tissue		21	46	6	71.2
Paracancer		9	50	9	86.7
Late group	68				
Tumor tissue		27	34	7	56.2^ab^
Paracancer		8	48	12	88.2

**Note:** a compared with paracancerous tissue, *p* < 0.5; b compared with early colon cancer, *p* < 0.05. “—” stands for negative expression, “±” represents expressions not significantly differentiated with adjacent normal tissue, and “++” stands for expression significantly higher than adjacent normal tissue.

**Figure 3:** Survival analysis on patients with colon tissues expressing high and low content of IL-35 X axis represents survival days and y axis indicates percentage of survival.

### IL-35 suppresses colon cancer

The results showed that the total RNA of Colon26 and Colon26/IL-35 cells had bright and clear bands at 18S and 28S, and the width of the 28S was almost equal to 18S [17]. Total RNA Colon26 and Colon26/IL-35 cells were electrophoresed with ethidium bromide. IL-35 DNA was quantitated by RT-PCR. RT-PCR product of Colon26/IL-35 cells formed a specific band near 434bp (Figure 4), while the RT-PCR product of Colon26 cells had no specific band formation, indicating that Colon26/IL-35 cell line had stable expression of IL-35 mRNA as opposed to Colon26 cell line. Semi-quantitative analysis of Gel.33 was used to select the NO.3 cell clone with relatively high expression level of IL-35 as the object of follow-up study.

**Figure 4:** RT-PCR product of Colon26 and Colon26/IL-35 cell lines **(A)** the image of the RT-PCR product of Colon26 and Colon26/IL-35 cell lines; **(B)** the statistic bar graph of the RT-PCR product of Colon26 and Colon26/IL-35 cell lines in (A).

In *in vivo* experiments (Colon26/IL-35 cell line), the tumor formation was gradually evident at the right paw pad of the mice (Figure 5A). When the average tumor volume was 0.8 cm^3^, the tumor growth has stagnated and then subsided. The control group (Colon26 cell line) was under continuous growth. The mean values of tumor volume changes were calculated for each group (Figure 5B). On day 25 after innoculation, the tumor volume of the experimental group and the control group were 0.22 ± 0.09 cm^3^ and 1.17 ± 0.53 cm^3^, respectively. The tumor volume of mice in the experimental group was significantly lower than that in the control group (p=0.0273).

**Figure 5:** **(A)** Photographs of representative mice and tumors. **(B)** Changes in tumor volume after transplantation of Colon26 and Colon26/IL-35 cell lines. X axis represents days after transduction of vector containing Colon26 into mice. Colon26: transduction with empty vector containing Colon26; Colon26/IL-35: transduction with Colon26 cell line carrying pCAGSIH cloned with IL-35 cDNA.

### IL-35 inhibits β-catenin expression in colon cancer cells

Wnt/β-catenin signaling pathway is highly involved in the maintennance of potency to differentiate in stem cells, while abnormally overactivated Wnt signaling has been found in colon cancer [18]. To examine the effect of IL-35 in Wnt signaling pathway, the expression of β-catenin, an important component of canonical pathway, in Colon26/IL-35 and Colon26 cells was analyzed. Both mRNA and protein levels of β-catenin were suppressed by rhIL-35 (Figure 6). Furthermore, the nuclear translocation of β-catenin was also reduced by IL-35 [19]. To further confirm the correlation between IL-35 and β-catenin signaling pathway, we transfected the Colon26/IL-35 and Colon26 cells with plasmids overexpressing IL-35, β-catenin or combination of them. Compared with the control group, the effects of IL-35 on cell proliferation, migration, invasion, apoptosis and cancer stem cells were abolished in β-catenin overexpressing cells. These data demonstrated that IL-35 might inhibit colon cancer cells via β-catenin pathway.

**Figure 6:** The protein level of β-catenin was measured by western blotting. Colon26/IL-35 and Colon26 cells were treated with 100 ng/mL rhIL-35. n = 3 ^*^P < 0.05.

Similarly, we measured the β-catenin expression level in colon cancer tissues of patients, which were divided into metastasis group and non-metastasis group. RT-qPCR was used to determined the mRNA of *CTNNB1*. β-catenin is more abundant in the tumor tissues residing in patients with lymph node metastasis (Figure 7, p=0.0178). The immunohistochemical results showed consistency with the expression level measured by RT-qPCR (Figure 8).

**Figure 7:** The relative expression of β-catenin in colon cancer tissues of patients with or without lymph node metastasis

**Figure 8:** Immunohistochemistry of β-catenin in colon cancer tissues of patients with or without metastasis (SP, ×200) **(A)** The expression of β-catenin in colon cancer tissue of patients without lymph node metastasis; **(B)** The expression of β-catenin in colon cancer tissue of patients with lymph node metastasis.

## DISCUSSIONS

With the improvement of people’s living standards and the improvement of dietary structure, the incidence of colon cancer increased year by year. On the other hand, the traditional surgery, radiotherapy and chemotherapy and other major treatment of colon cancer still failed to significantly improve the survival rate of colon cancer over the years. Recent years has witnessed the deepened understanding of tumor immunology, making the pathogenesis of colon cancer has been further clear [20, 21]. Tumor is the product of normal cell undergoing malignant transformation, and theoretically cancer cells with various antigens are different from normal cells, which could activate immune response specific for them. However, under some circumstances, such as immunodeficiency, the immune system is not potent enough to combat the growth of cancer cells, which foster their proliferation, and extensive migration [22]. Therefore, a comprehensive enhancement of the immune status of patients can employ the immune mechanism to combat cancers, and will attract more and more attention by the majority of clinicians [23, 24]. IL-35 is a new member of the γc family and contains four helix cytokine domains with IL-2, IL-12, IL-15 and IL-18, all of which pathway through γc the chain transducts the signal into the cell and exert anti-tumor effects thereby. These cytokines are highly homologous [25].

IL-35 is an important inflammatory cytokine, which is critical for regulating tissue damage and immune response [26]. IL-35 is associated with a variety of malignancies and is a promising tumor marker. The results showed that IL-35 expression in tumor tissue of colon cancer patients increased, and almost no expression in adjacent tissues, suggesting that IL-35 may be implicated in regulating the proliferation of tumor cells [27]. The results showed that colon cancer tumor tissue could secrete IL-35, though its role in tumor formation, promote tumor growth is elusive. The high expression of IL-35 in colon cancer tissue is involved in the regulation of monocyte-macrophage and neutrophil killing. IL-35 can promote tissue catabolism, and fat, protein degradation, may be involved in the occurrence of cancer cachexia [28].

Tumor is heterogeneous that not all tumor cells have invasion and metastasis ability, but only some special subgroups have metastatic potential. In addition, the respective metastatic potentials of those metastatic potential subpopulation of tumor cells are also inconsistent [29]. Taking acount of various factors on the host, the difference in the outcome of the final subgroup of tumor cells will be more pronounced [30]. Therefore, tumor cells isolated from tissues other than tumor have different characteristics than primary tumor cells, due to their high potency of migration and abnormal proliferation. The colon cancer-like metastatic cells remainning in the tissue can simulate the residual tumor cells in colon cancer and the biological behavior of tumor cells that have metastasized. These cells can serve to establish lymph node metastasis model and be used to verify the therapeutic role of different treatment factors in postoperative lymph node metastasis of colon cancer.

It is worth noting that the role of cytokines is like a double-edged sword. On one hand, it can enhance the body’s immune function and kill tumor cells to maintain the health of the human body. On the other hand, the imbalance between cytokines will also cause a strong immune response to human body by bringing unexpected damage [31]. Clinical application of large doses of exogenous IL-2 to inhibit the growth of malignant tumors, which has a certain probability of producing undesired side effects, such as fever, nausea, muscle soreness, and some individual cases, so it’s necessary to stop treatment in time [32]. Transgenic therapy is performed by use of viruses or other methods to stimulate the immune function of the gene (such as IL-35 etc.) implanted tumor cells. After the success of gene transfer, the target gene will be replicated with the tumor cell division and proliferation, then continue to copy the expression, which sustained a constant secretion of a large number of immune cytokines, improving the immunity of the body. The results of this study showed that the colon cancer cells transfected with IL-35 gene could continue to proliferate and replicate along with the tumor cell proliferation at the early stage of inoculation, leading to abundant IL-35 protein synthesis and secretion, and then stimulate the comprehensive anti-tumor immunity. The effect of IL-35 on the relative lack of IL-35 synthesis cannot effectively inhibit the proliferation of colon cancer cells, tumor growth, the final occurrence of metastasis or death.

## MATERIALS AND METHODS

### Patients

A total of 141 patients with colon cancer who underwent surgical treatment from March 2004 to October 2007 were randomly selected from 73 males and 68 females aged 32 to 83 years with a median age of 56.2 years. Pathology confirmed that the patients including 42 cases of ascending colon, 14 cases of transverse colon, 25cases of descending colon, 60 cases of sigmoid colon, 16 cases of Dukes A in clinical stage, 55 cases of Dukes B, 52 cases of Dukes C, 18 cases of Dukes D; Duke stage A was regarded as early stage, Stage B and C were regarded as middle stage, and Stage D was redefined as late stageThose patients do not have a history of other cancers, or synchronous multiple cancers, never chemotherapy or radiotherapy before the tumor tissues and adjacent normal tissues were sampled. Whole blood samples weree derived from colon cancer patients at the time of diagnosis. Written informed consents were obtained from patients followed by approval from Ethical Committee of Medical college, Nanjing university. Whole blood was separated into serum and cellular fractions within 2 h after blook was derived. For serum RNA isolation, equal volume of Trizol was used, and three steps of phenol/chloroform purification were added since serum is full of proteins.

### Preparation of cell lines Colon26/IL-35

Colon 26 cell lines were cultured in Dulbecco’s modified Eagle’s medium (DMEM) supplemented with 10% fetal bovine serum, penicillin (100 U/ml), streptomycin (100μg/ml), and a 7% CO_2_ environment. Early-passage cell lines were used for studies. Murine IL-35 gene was cloned into the pCAGSIH expression plasmid. Colon26 cells were stably transfected by using the Lipofectamine Plus reagent (Invitrogen) and clones of cells showing stable transfection were obtained by antibiotic resistance selection using G418 (Gibco, Grand Island, NY, USA) and hygromycin-B (Sigma, St Louis, MO, USA).

### Animal assays

Forty-eight BALB/c mice, female, 6-8w, weight 25±2g, purchased from the experimental animal center, certificate number: DK0408-0041. Colon26 cell line, a poorly differentiated adenocarcinoma of the colon, was donated by the research center. Retroviral vectors carrying IL-35 cDNA LXSN, ecotropic ψ2 packaging cells and amphotropic PA317 packaging cells were donated by the Chiba Cancer Center, Japan.

Nude mice were randomly allocated into control and IL-35 overexpressing group, and anesthetized with methoxyfluorance by inhalation. The abdomen was prepared for sterile surgery. A small abdominal incision was made, and the cecum identified and isolated between scrips of sterile gauze. About 5×10^6^ viable tumor cells in 0.1ml serum-free medium were injected into the cecal wall from the serosal side. Cells were injected in a way that they infiltrate between submucosal and subcerosal tissues. After 6 weeks animals were sacrificed by cervical dislocation and abdominal organs were examined and extracted. All experimental procedures involving animals were in accordance with the Guide for the Care and Use of Laboratory Animals (NIH publication nos. 80-23, revised 1996) and were performed in compliance with the institutional ethical guidelines for animal experimentation.

### RNA extraction and real-time polymerase chain reaction (RT-PCR)

Total RNA from colon cancer samples was extracted with RNAiso Plus (Takara, Dalian, China), and cDNA synthesized with the PrimeScript RT reagent Kit (Takara, Dalian, China). Quantitative PCR was performed using a SYBR Premix Ex TaqTM II (Takara, Dalian, China). Data were collected on an ABI StepOne real-time PCR system (Applied Biosystems, Carlsbad, CA). The expression level of IL-35 were normalized to the housekeeping gene Gapdh (ΔCt), and the results were calculated with 2^-ΔΔ^Ctt method.

### Western blotting

Colon cancer samples were harvested with RIPA lysis buffer (P0013; Beyotime, Shanghai, China). Proteins were denatured in 1×SDS loading buffer, boiled, and run on denaturing gels. Proteins were transferred onto PVDF membranes (Millipore, Billerica, Massachusetts) at 300 mA. After blocking in 5% BSA for 1 h, membranes were incubated in primary antibodies with 2% BSA overnight at 4 °C followed by HRP-conjugated secondary antibodies for 1 h at room temperature. Anti-human IL-12p35 antibodies, anti-β-catenin antibodies (Santa Cruz Biotechnology, USA), anti-GAPDH (1:10000; Boster, Wuhan, China) were used. Specific proteins were detected with enhanced chemiluminescence (BioRad, Hercules, CA, USA) and images of the blots were obtained using the ImageQuant LAS 4000 mini system (GE healthcare, London, U.K.).

### Immunohistochemistry

Formalin-fixed, paraffin-embedded (FFPE) surgical specimens obtained from patients were used for immunohistochemical staining. After deparaffinization, the specimens were rehydrated in graded ethanol (100, 95, 70, and 50%) and processed using labeled streptavidin-biotin-peroxidase method. Heating in citrate buffer (pH 6.0) for 5 minutes, the antigen was retrieved. After blocking by endogenous peroxide with 3% H_2_O_2_ in methanol for 5 min, washes with phosphate-buffered saline (PBS), and reblocking with blocking serum for 30 min, slides were incubted with anti-human IL-12p35 antibodies or anti-β-catenin depending on the experiments (Santa Cruz Biotechnology, USA) at 4°C overnight, and then incubated with biotin-labelled secondary antibodies at 30°C for 50 min. IL-35 expression was rated as negative (no positive staining), low (less than 30% cells were stained) and high (more than 30% cells were stained).

### Enzyme-linked immunoassay (ELISA)

The protein level of IL-35 was detected in culture supernatants and tumor homogenate using human IL-35 ELISA kit (AdipoGen AG, Liestal, Switzerland) according to the manufacturer’s instructions [33]. All samples were assayed in triplicate.

### Statistical analysis

Data were expressed as mean (± SE) and analyzed by a SPSS software package (SPSS Standard version 13.0, SPSS Inc, USA). Differences between variables were assessed by the Chi-square test. Survival analysis of patients with colon cancer was calculated by Kaplan-Meier analysis. Survival time was calculated from the date of surgery until either death, the termination date of the study, or the last date of contact for patients who were still alive at the end of the study. Unpaired Student’s t test and one way ANOVA were used to assess the statistical significant of difference. P values under 0.05 were considered statistically significant.

## CONCLUSIONS

IL-35 is an indicator of cellular immune function, which can promote the secretion of IFN-γ and can produce anti-tumor effect synergistically. In colon cancer patients, IL-35 and IFN-γ production are closely related. The correlation between the two studies showed that there was no gender difference in the two cytokines, but with the increase of the patient’s age, the tumor volume increased, the tumor tissue infiltration increased, the disease was late or the merger of lymph node metastasis, serum IL-35 Of the level of performance is relatively insufficient, the use of gene immunization technology to improve its secretion level, may become a powerful means of adjuvant treatment of colon cancer in the future. The IL-35 gene was implanted into Colon26 cells by retroviral vector gene transfer technique, which was characterized by high secretion of IL-35 by cloning and screening. This transfer can further induce tumor-bearing mice anti-tumor immune response by increasing the body INF-γ content, increasing the expression of MHC molecules on the cell surface and strengthening the CTL effect of cytotoxic T cells and other cellular immune mechanism inhibition of colonic tumor growth. In addition, the body’s specific immune mechanism can effectively inhibit lymph node metastasis of colon cancer cells. Its role in the removal of colon cancer after the remaining residual tumor cells and preventing the metastasis and recurrence of colon cancer has far-reaching significance.
